# Ground Movement Analysis Based on Stochastic Medium Theory

**DOI:** 10.1155/2014/702561

**Published:** 2014-02-18

**Authors:** Meng Fei, Wu Li-chun, Zhang Jia-sheng, Deng Guo-dong, Ni Zhi-hui

**Affiliations:** ^1^School of Civil Engineering, Central South University, Changsha 410075, China; ^2^Chongqing Education University, Chongqing 400067, China; ^3^Key Laboratory of Hydraulic and Waterway Engineering of the Ministry of Education and National Engineering Research Center for Inland Waterway Regulation, Chongqing Jiaotong University, Chongqing 400074, China

## Abstract

In order to calculate the ground movement induced by displacement piles driven into horizontal layered strata, an axisymmetric model was built and then the vertical and horizontal ground movement functions were deduced using stochastic medium theory. Results show that the vertical ground movement obeys normal distribution function, while the horizontal ground movement is an exponential function. Utilizing field measured data, parameters of these functions can be obtained by back analysis, and an example was employed to verify this model. Result shows that stochastic medium theory is suitable for calculating the ground movement in pile driving, and there is no need to consider the constitutive model of soil or contact between pile and soil. This method is applicable in practice.

## 1. Introduction

Displacement piles are widely used in pile foundation engineering and ground treatment. During the driving process of displacement piles, the lateral expansion and uplift of surrounding soil may have significant effect on adjacent buildings, underground structures, and municipal pipelines. It is an important issue in geotechnical engineering.

At present, methods which are widely used in compaction effect analysis of displacement piles are cylindrical cavity expansion method, spherical cavity expansion method, and strain path method. Cylindrical cavity expansion method [1–6] assumes that the initial holes are cylindrical with infinite length, and the pile driving process is equivalent to the expansion process of the cylindrical cavity. Then the three-dimensional problem is simplified to a plane strain problem, which makes it impossible to solve ground movement. Spherical cavity expansion method assumes that the initial holes are spherical, and the soil is simplified to infinite space or semi-infinite space [7–13]. But this method is only applicable to homogeneous soil, and boundary condition of the semi-infinite space's surface is complicated. Strain path method was proposed by Baligh et al. [14–18]. It overcomes the shortcoming that the cavity expansion theory does not consider the impact of depth. An independent strain field is obtained by analyzing the process of a smooth, round pile driven into soil. Owing to the fact that the rotation of soil units and the surface effect of ground are neglected, this method is also unable to calculate the ground movement. Numerical analyses are widely used in the calculation of soil deformation [19–23], but their accuracy depends highly on the stress-strain relationships and parameters of soil and pile-soil interface.

Stochastic medium theory was initially proposed by the Polish scholar Litwiniszyn, and then it was developed by Bao-chen et al. [24–28]. Compared with mechanical analysis method, stochastic medium theory does not need constitutive model of rock or soil and its mechanical parameters. At present, stochastic medium theory is mainly used to calculate ground movement caused by mining, tunnel construction, and so on, which is convergent movement caused by excavation of underground space. While in the process of pile driving, soil is vertically and radially compacted, and the ground movement is mainly expanding movement—a process with same property but opposite direction.

In this paper, the problem of pile driving into transverse isotropy layered soil is simplified to an axisymmetric problem. Then vertical and horizontal ground movement functions are obtained using stochastic medium theory, and ground movement parameters are calculated by back analysis. At last, an engineering example is also presented to verify the theoretical answer.

## 2. Calculation Model of Ground Movement

### 2.1. Introduction to the Stochastic Medium Theory

In an Euclidean space where *z* is the vertical coordinate and *x* and *y* are orthogonal horizontal coordinates, according to the movement transfer process of medium, the vertical movement function *W*(*z*, *x*, *y*) in depth *z* is subjected to

(1) ∂W(z,x,y)∂z=B11(z,x,y)∂2W(z,x,y)∂x2 +B12(z,x,y)∂2W(z,x,y)∂x∂y +B22(z,x,y)∂2W(z,x,y)∂y2 +A1(z,x,y)∂W(z,x,y)∂x +A2(z,x,y)∂W(z,x,y)∂y +N(z,x,y)W(z,x,y),

where *B*_11_, *B*_12_, *B*_22_, *A*_1_, *A*_2_, and *N* are parameters determined by the properties of medium. Equation (1) is similar to the Kolmogorov equation in continuous stochastic process, so medium which satisfies (1) is named as stochastic medium, such as soil, sand, and rock.

If the unit vertical movement *W*_*e*_ caused by excavation of a 1 × 1 × 1 space underground at a depth *H* (as shown in Figure 1) can be obtained, vertical movements induced by excavation of any other shapes can be calculated through integration. The unit vertical movement function can be solved as in Figure 1.

In a local coordinate system (*z*_*e*_, *x*_*e*_, *y*_*e*_), of which origin is the center of the unit, according to the boundary conditions, the unit vertical movement function is the solution of

(2) ∂We∂ze=LWe,We|ze=0={1,−12≤xe≤12,−12≤ye≤120,other=δ(xe,ye),

where *L* = *B*_11_(∂^2^/∂*x*_*e*_^2^) + *B*_12_(∂^2^/∂*x*_*e*_∂*y*_*e*_)+⋯, *δ*(*x*_*e*_, *y*_*e*_) is the Dirac function.

For typical transverse isotropy layered soil, (2) can be simplified to

(3) $$\begin{array}{c} \frac{\partial W_{e}}{\partial z_{e}}=B\left(z_{e}\right)\left(\frac{\partial^{2}W_{e}}{\partial x_{e}^{2}}+\frac{\partial^{2}W_{e}}{\partial y_{e}^{2}}\right),\\ W_{e}{|}_{z_{e}=0}=\delta \left(x_{e},y_{e}\right). \end{array}$$

If the volume of soil remains the same during deformation process (a coefficient will be introduced afterwards to take the deformation of soil into account), it can be deduced that vertical displacement *W*_*e*_ and horizontal displacement *U*_*ex*_, *U*_*ey*_ satisfy

(4) $$\begin{array}{c} \frac{\partial W_{e}}{\partial z}+\frac{\partial U_{ex}}{\partial x}+\frac{\partial U_{ey}}{\partial y}=0. \end{array}$$

Assuming the displacement vector of soil point to the center of the unit, from (3) and (4), the movement of layered soil caused by unit excavation can be acquired as

(5) $$\begin{array}{c} W_{e}=\frac{1}{r^{2}\left(z_{e}\right)}\exp\frac{-\pi \left(x_{e}^{2}+y_{e}^{2}\right)}{r^{2}\left(z_{e}\right)},\\ U_{ex}=\frac{x_{e}}{r\left(z_{e}\right)}\frac{dr\left(z_{e}\right)}{dz_{e}}W_{e},\\ U_{ey}=\frac{y_{e}}{r\left(z_{e}\right)}\frac{dr\left(z_{e}\right)}{dz_{e}}W_{e}, \end{array}$$

where *r*(*z*_*e*_) is influence radius at different depths, *r* ^2^(*z*_*e*_) = 4*π*∫_0_^*z*_*e*_^ *B*(*z*_*e*_)*dz*_*e*_.

### 2.2. Calculation Model

The process of driving a pile into horizontally layered soil can be simplified to an axisymmetric problem. Then, (5) can be expressed as below in cylindrical coordinates (*z*_*e*_, *ρ*_*e*_, *θ*_*e*_):

(6) We(ρe)=1r2(ze)exp⁡(−π(xe2+ye2)r2(ze))=1r2(ze)exp⁡−πρe2r2(ze),Ue(ρe)=Uex2+Uey2=ρer(ze)dr(ze)dzeWe=ρer3(ze)dr(ze)dzeexp⁡−πρe2r2(ze).

The influence radius *r*(*z*_*e*_) is a complex function without specific function. A parameter—influence angle *β*(*z*_*e*_)—can be defined as

(7) $$\begin{array}{c} \tan\beta \left(z_{e}\right)=\frac{z_{e}}{r\left(z_{e}\right)}. \end{array}$$

*β*(*z*_*e*_) reflects the mechanical property of overlying soil. At ground surface, *β*(*z*_*e*_) is a constant *β*(*H*), hereinafter abbreviated as *β*.

In order to calculate the horizontal movement at ground, another parameter—horizontal movement coefficient *b*—was defined, and for ground surface,

(8) $$\begin{array}{c} {\left[\frac{dr\left(z_{e}\right)}{dz_{e}}\right]}_{z_{e}=H}=2\pi b. \end{array}$$

In pile driving, the compaction process of soil is equivalent to the expansion process of a series of zero-volume units along the pile axis [7]. Supposing the pile's cross-section area at depth *z* is *A*(*z*), the volume of a micro unit will change from 0 to *A*(*z*)*dz*. As shown in Figure 2, when a pile whose length is *l* is driven into soil, the ground movement can be expressed as

(9) $$\begin{array}{c} F=\int_{0}^{l}F_{e}A\left(z\right)dz, \end{array}$$

where **F** is ground movement vector, **F** = (*W*, *U*). **F**_*e*_ is ground movement vector caused by unit excavation, **F**_*e*_ = (*W*_*e*_, *U*_*e*_).

In order to take the compaction of soil into consideration, a compaction coefficient *η* was defined. Then (9) can be modified to

(10) $$\begin{array}{c} F=\eta \int_{0}^{l}F_{e}A\left(z\right)dz. \end{array}$$

For piles with constant cross-section area *A*, the ground movement in pile driving can be deduced from (7), (8) and (10):

(11) W(ρ)=η∫0lAWe dz=ηA tan2 β∫0l1z2exp⁡(−πρ2 tan2 βz2)dz=ηA tan βρ[1−Φ(2πρtan βl)],U(ρ)=η∫0lAUe dz=2η tan3 βπAbρ∫0l1z3exp⁡(−πρ2 tan2 βz2)dz=bηA tan βρexp⁡(−πρ2 tan2 βl2),

where *ρ* is the distance from calculation point to the center of pile. Φ(*x*) is the distribution function of standard normal distribution.

### 2.3. Parameters' Determination

There are three parameters in the calculation model, respectively, influence angle *β*, horizontal movement coefficient *b*, and compaction coefficient *η*, which can be expressed as a vector **X**, **X** = {*β*, *b*, *η*}. The ground movement can be calculated after **X** was obtained from observational data using back analysis method.

If *W*_i_*, *U*_i_* represent a series of ground movement observational data, and *W*_*i*_, *U*_*i*_ are corresponding calculated data based on parameter **X**, according to least square method, their consistency can be assessed by

(12) $$\begin{array}{c} R\left(X\right)=\sum {\left(W_{i}-W_{i}^{*}\right)}^{2}+\sum {\left(U_{i}-U_{i}^{*}\right)}^{2}. \end{array}$$

The less the *R*(**X**) is, the better the parameter **X** is. To find the best ground movement parameters through back analysis is to find a set of **X** ∈ **R** ^3^ which makes

(13) $$\begin{array}{c} R\left(X\right)=\min\left\{\sum {\left(W_{i}-W_{i}^{*}\right)}^{2}+\sum {\left(U_{i}-U_{i}^{*}\right)}^{2}\right\}. \end{array}$$

This is an unconstrained optimization problem. In this paper, a program PAFI written by Visual Basic was used to find the best ground movement parameters. Then the relative ground movement can be obtained by (11).

## 3. Engineering Example

In order to verify the calculation model and program, results of the in situ test conducted by Hwang et al. [29] are employed in this paper. Test pile is a precast concrete pile whose diameter *d* is 800 mm and length *l* is 34 m. From the ground surface to the depth of 40 m, the strata are, respectively, layers of yellow clays with organic materials (0~3 m), gray silty sands (3~8 m), soft clays (8~12 m), medium-dense sands (12~21 m), a clay layer interbedded with some thin layers of fine sand (21~32 m), and medium-to-dense sands (32~40 m) [29]. Locations of ground movement monitoring points are shown in Figure 3. Three inclinometer tubes are laid, respectively, at distances of 3*d*, 6*d*, and 9*d* from the centre of the pile. Nine settlement marks are located at different positions on one line.

In the test, ground movement was measured when the pile was driven in 9 m, 17 m, 25 m, and 34 m. Monitoring results of ground movement induced by pile driving are shown in Figures 4 and 5. Using the test results, back analysis conducted by PAFI program shows that influence angle *β* = 0.222 rad, horizontal movement coefficient *b* = 0.353, and compaction coefficient *η* = 0.601. Then ground movement can be obtained by (11). Their comparison with measured results is also shown in Figures 4 and 5. As can be seen, calculated results agree well with observational data, which means this method has good applicability.

## 4. Conclusions

For horizontally layered soil, ground movement in pile driving was calculated by stochastic medium theory.

1. The pile driving process was simplified to an axisymmetric problem. Then the vertical and horizontal ground movement functions are derived. The vertical ground movement is a normal distribution function, and the horizontal ground movement is an exponential function.
2. There are three parameters in the calculation model, respectively, influence angle *β*, horizontal movement coefficient *b*, and compaction coefficient *η*. They can be obtained from observational data using back analysis.
3. Analysis of an engineering examples shows that this method is applicable to compute surface movement caused by pile driving. Stochastic medium theory does not need to consider the constitutive model of soil or pile-soil interface, so it is easier to be applied in practice.

## Figures and Tables

**Figure 1:** Calculation model for unit excavation.

**Figure 2:** Integral domain in pile driving.

**Figure 3:** Positions of ground movement monitoring points.

**Figure 4:** Observational data and calculated results of vertical movement.

**Figure 5:** Observational data and calculated results of horizontal movement.
